# Mechanisms Underlying the Differences in the Pharmacokinetics of Six Active Constituents of Huangqi Liuyi Decoction between Normal and Diabetic Nephropathy Mouse Models

**DOI:** 10.1155/2022/2481654

**Published:** 2022-10-15

**Authors:** Qun Wang, Yonglin Wang, Wen Liu, Dingyan Lu, Yang Jin, Nian Tang, Ya Shi, Zipeng Gong, Weiyi Tian, Ting Liu

**Affiliations:** ^1^Guizhou University of Traditional Chinese Medicine, Huaxi University Town, Guiyang 550025, China; ^2^Guizhou Provincial Key Laboratory of Pharmaceutics, Guizhou Medical University, Beijing Road, Guiyang 550004, China

## Abstract

The aim of this study was to explore the mechanisms underlying the differences in the pharmacokinetics of Huangqi Liuyi decoction extract (HQD) under physiological and pathological conditions. The roles of liver cytochrome P450 metabolic enzymes (Cyp450) and small intestinal transporters were also investigated. The cocktail probe drug method was used to investigate the effects of diabetic nephropathy (DN) and HQD on metabolic enzyme activity. The expression levels of liver Cyp450 metabolic enzymes (Cyp1A2, Cyp2C37, Cyp3A11, Cyp2E1, and Cyp2C11) and small intestinal transporters (breast cancer resistance protein (BCRP), P-glycoprotein (P-gp), organic cation transporters (OCTs), and multidrug resistance-associated protein (MRPs) were determined using western blot. Compared to normal mice, the expression of OCT1, OCT2, MRP1, and MRP2 was increased in DN mice, while that of P-gp and BCRP (*P* < 0.05 and *P* < 0.001) was inhibited. HQD inhibited expression of Cyp1A2 and Cyp3A11 and increased the expression of P-gp and BCRP in normal mice. In DN mice, HQD induced expression of BCRP and inhibited expression of Cyp2C37, Cyp3A11, OCT2, MRP1, and MRP2. The activity of each Cyp450 enzyme was consistent with changes in expression. The changes in pharmacokinetic parameters of HQD in DN might, in part, be secondary to decreased expression of P-gp and BCRP. HQD varied in regulating transporter activities between health and disease. These findings support careful application of HQD-based treatment in DN, especially in combination with other drugs.

## 1. Introduction

Diabetic nephropathy (DN), one of the most serious complications of diabetes mellitus, is characterized by proteinuria, microalbuminuria, increased blood pressure, and a continuous decline in the glomerular filtration rate [1–3]. Most cases progress to end-stage renal disease [4]. Prevention or early treatment of DN may improve patient survival and quality of life and lower medical costs [5]. Due to their limited side effects and toxicity, traditional Chinese medicines (TCMs) are widely applied in the treatment of diseases [6] including diabetic complications [7, 8]. Huangqi Liuyi decoction, which is composed of *Radix Astragalus* and *Radix Glycyrrhizae*, has been used in China since the Song dynasty. (A.D. 960 to 1279 A.D.). *Astragalus* inhibited the formation of renal interstitial fibrosis and slowed down the development of DN. *Glycyrrhizae* decreased fasting bloodglucose and antirenal oxidative stress [9, 10]. Huangqi Liuyi decoction significantly inhibited glucose reabsorption in renal tubular epithelial cells, decreasing the fasting blood glucose and limiting renal fibrosis in DN rats [11, 12]. In pilot studies [13], we found that several ingredients found in the Huangqi Liuyi decoction, namely, astragalus saponin, astragalus flavone, astragalus polysaccharide, and glycyrrhizic acid (AKA HQD), delayed the development of DN in db/db mice when combined. HQD could significantly decrease the fasting blood glucose (FBG), 24 h urinary protein (24 h U-Alb), urea nitrogen (BUN) serum creatinine (Scr), and triglyceride (TG) in DN mice (*P* < 0.05). Moreover, there were no significant differences in pharmacodynamics between HQD and Huangqi Liuyi decoction. Furthermore, following oral administration of HQD, the area under the curve (AUC) of the six active ingredients (astragaloside IV, calycosin-7-O-*β*-D-glucoside, calycosin-glucuronide, ononin, formononetin, and glycyrrhizic acid) and the *C*_max_ values of astragaloside IV, ononin, and formononetin in DN mice were increased (*P* < 0.05), while the CL_Z/F_ (clearance rate) had slowed (*P* < 0.05).

Changes in the pharmacokinetics of drugs *in vivo* under pathological conditions may be caused by alterations in drug metabolic enzymes and transporters [14, 15]. Liver CYP450 enzyme is involved in the metabolism of approximately 90% of clinical drugs. CYP450 enzyme metabolism is linked to 70% of drug-drug interactions [16]. In the liver, TCMs can inhibit or induce CYP450 enzymes and alter drug effects or, when used in combination with other drugs, and promote toxicity [17]. Numerous drug transporters found on intestinal epithelial cells are targets to improve drug absorption and bioavailability [18]. Uptake transporters (organic cation transporters, OCTs) are involved in the transport of approximately 40% of clinical drugs [19]. In addition to uptake transporters, P-glycoprotein (P-gp), breast cancer resistance protein (BCRP), and multidrug resistance-associated protein (MRP) as intestinal efflux transporters, actively transport many endogenous substances and drugs from enterocytes to the intestinal lumen or the systemic circulation. Flavonoids are mainly absorbed in the intestine, and this efflux effect can significantly affect the bioavailability of flavonoids, and consequently, their clinical efficacy [20]. Moreover, under pathological conditions, a certain index component of a TCM may change the absorption and metabolism of other drugs by inducing or inhibiting the expression of metabolic enzymes and transporters. This, in turn, alters the drug plasma concentration and efficacy [21]. Herein, HQD-mediated changes in Cyp450 enzyme and transporter (BCRP, P-gp, OCT, and MRP) expression and activity under physiological and pathological conditions were assessed to clarify the differential pharmacokinetic mechanisms of six active ingredients in HQD between normal and DN mouse models.

## 2. Materials and Methods

### 2.1. Materials

The following reference substances were employed: astragaloside IV (purity > 99.0%), calycosin-7-O-*β*-D-glucoside (purity > 98.0%), calycosin-glucuronide (purity > 98.0%), formononetin (purity > 98.0%), ononin (purity > 98.0%), and glycyrrhizic acid (purity > 99.0%). Puerarin (IS, purity > 98.0%) and digoxin (IS, purity > 98.0%) were obtained from the National Institute for the Control of Pharmaceutical and Biological Products (Beijing, China).

Testosterone (D1509G72399) and acetaminophen (B14A9E58584) were obtained from Shanghai Yuanye Bio-Technology Co., Ltd. (Shanghai, China); omeprazole (Y1306C4251), aglicem (Y08M8C0197), and chlorzoxazone (Y07M7C14306) were obtained from Suzhou Meilun Biotechnology Co., Ltd. (Suzhou, China); dextrorphan (JC0496-201606111) was obtained from Shanghai Jianchao Bio-Technology Co., Ltd. (Shanghai, China); hydroxytolbutamide (IS10603-10M), 5-hydroxyomeprazole (IS10787), 6-hydroxychloroxazone (IST000286), and 6*β*-hydroxytestosterone (FN02261502) were obtained from A ChemTek Inc. (Worcester, MA, USA); and acetonitrile and methanol were purchased from Merck KGaA (Darmstadt, Germany). All other chemicals used were of analytical grade. The bicinchoninic acid (BCA) protein assay kit was obtained from Shanghai Solarbio Bioscience & Technology Co., Ltd (Shanghai, China); the membrane protein extraction kit, goat antimouse immunoglobulin G (31430), and goat antirabbit (31460) were obtained from Thermo Fisher Scientific (Waltham, MA, USA); and anti-OCT1 (ab178869), anti-OCT2 (ab179808), anti-MRP1 (ab32574), anti-MRP2 (ab203397), anti-BCRP (ab207732), anti-P-gp (ab170904), anti-1A2 (ab22717), anti-2C9 (ab4236), anti-2C19 (ab137015), anti-2E1 (ab28146), and anti-3A4 (ab3572) were obtained from Abcam (Cambridge, England).

We first determined the preparation process of astragalus saponins, astragalus flavones, astragalus polysaccharides, and glycyrrhizic acid extract. To this end, we prepared astragalus saponins and astragalus flavones extract using a macroporus resin column; astragalus polysaccharides extract was prepared using water extraction and alcohol precipitation; and glycyrrhizic acid extract was prepared using acid precipitation. The extract content of each component extracted from the three batches of Astragalus and Glycyrrhizae is shown in Table 1.

According to the ratio of Huagqi Liuyi decoction (6 : 1, *Astragalus* : *Glycyrrhiza*), processing 18 kg of *Astragalus* and 3 kg of *Glycyrrhiza* yielded 115.38 g of astragalus saponins (72.04%, including 2.69% of astragaloside IV), 44.64 g of astragalus flavone (69.43%, including 1.62% of calycosin-7-O-*β*-D-glucoside, 1.42% of calycosin-glucuronide, 0.89% of ononin, 0.31% of formononetin), 279.36 g astragalus polysaccharides (65.82%), and 32.01 g glycyrrhizic acid (82.04%). The dry extract of astragalus saponins, astragalus flavones, astragalus polysaccharides, and glycyrrhizic acid was mixed together, and the HQD samples needed for this experiment were obtained. The high performance liquid chromatography-tandem mass spectrometry (HPLC-MS/MS) chromatogram of HQD is displayed in Figure 1. Puerarin and digoxin comprised the internal standard (IS). The HPLC-MS/MS chromatogram of the six reference substances (astragaloside IV, calycosin-7-O-*β*-D-glucoside, calycosin- glucuronide, ononin, formononetin, and glycyrrhizic acid) is shown in Figure 1(b), and the HQD sample is shown in Figure 1(c).

### 2.2. Animals

Ten-week-old db/db male mice and db/m mice were obtained from the Model Animal Research Center of Nanjing University (qualified number SCXK [Su] 2020–0018) and raised in a specific pathogen-free laboratory (SPF) of the Experimental Animal Center of Guizhou Medical University for 2 weeks. Ten-week-old db/db mice develop nephropathy at 12 weeks of age [22, 23]. All mice were housed in polypropylene cages and maintained under standard conditions, with a relative humidity of 60% ± 5%, and a light-dark cycle of 12 h. Animal studies complied with the European Community guidelines (EEC Directive of 1986; 86/609/EEC) and were approved by the Animal Ethical Committee of Guizhou Medical University (NO1702060).

### 2.3. Statistics

All data are presented as the mean ± standard deviation. Statistical analysis between the two groups was performed using the Statistical Package for the Social Sciences version 23 software program (IBM Corporation, Armonk, NY, USA). *P*-values <0.05 between the two groups were considered statistically different.

### 2.4. Preparation of Mouse Liver Microsomes

The mice were sacrificed 24 hours after the last dose of HQD. Livers were quickly removed and then washed three times with ice-cold 1.15% KCl solution. They were then weighed and homogenized with a tissue grinder at 4,000 rpm in an ice-cold water bath. The resulting sediment was then suspended in phosphate-buffered saline (PBS, pH 7.4) and centrifuged at 12,000 × *g* for 20 minutes at 4°C. The supernatant fraction was centrifuged again at 100,000 × *g* for 45 minutes at 4°C. Then, the supernatant was discarded, and the liver microsomes were suspended uniformly with Tris-HCl buffer (pH 7.4). The protein concentration of the liver microsomes was determined using a BCA kit. Microsomes were stored at −80°C until use.

### 2.5. Effects of DN and HQD on the Activity of Liver Metabolic Enzymes

Liver metabolic enzymes, including CYP1A2, 2C19, 3A4, 2E1, and 2C9, were used as the research objects. The cocktail probe substrate method is the most commonly used method for the determination of metabolic enzyme activity [24]. The specific probe substrates of Cyp450 isozymes were incubated with the liver microsomes of the control group, model group, control HQD-3d group (normal mice were orally administered HQD 0.96 g/kg once a day for 3 consecutive days), and model HQD-3d group (same oral administration as normal mice). The oral dose of HQD in mice was converted from the clinical dose for humans. The activity differences in major Cyp450 enzymes involved in drug metabolism among the different groups were evaluated by measuring the number of metabolites produced by specific probe substrates, and the effects of DN and HQD on Cyp450 enzyme activity in mice were characterized.

#### 2.5.1. Preparation of Mixed Probe Substrate Solutions

Mixed probe substrate solutions were prepared separately by dissolving phenacetin, omeprazole, testosterone, chlorzoxazone, and tolbutamide into methanol. These solutions were diluted with PBS (1 mM; pH, 7.0) to final concentrations of 150.0, 5.0, 2.5, 10.0, and 100.0 *μ*mol/L before use, and then preheated at 37°C for standby.

#### 2.5.2. Preparation of Mixed Probe Substrate Metabolite Solutions

Mixed probe substrate metabolite solutions were separately prepared by dissolving acetaminophen, 5-hydroxyomeprazole, 6*β*-hydroxytestosterone, 6-hydroxychlorzoxazone, 5-hydroxytolbutamide, and puerarin (IS) in methanol. These solutions were diluted with PBS (1 mM; pH, 7.0) to final concentrations of 102.1, 102.9, 100.2, 100.5, 99.6 *μ*g/mL, and 1 *μ*g/mL before use, and then preheated at 37°C for standby.

#### 2.5.3. Preparation of the Incubated Liver Microsome Samples *in Vitro*

The incubation system, with a total volume of 200 *μ*L, consisted of liver microsomes (50 *μ*L, 1 mg/mL), PBS (50 *μ*L; pH 7.0), mixed probe substrate (80 *μ*L total; with the concentrations of phenacetin, chlorzoxazone, omeprazole, tolbutamide, and testosterone being 100, 150, 25, 100, and 50 *μ*mol/L, respectively), and NADPH (20 *μ*L, 1 mmol/L). All incubation samples were conducted in triplicate. The mixed solution of liver microsomes and probe substrate was preincubated at 37°C for 5 minutes. Then, NADPH, which was incubated at 37°C for 5 minutes, was added to initiate the reaction, and the incubation was allowed to continue at 37°C for 60 minutes in a constant temperature oscillator. To end the reaction, 400 *μ*L of iced methanol containing the IS (puerarin, 1 *μ*g/mL) was added. The samples were vortexed for 1 minute and centrifuged for 10 minutes (15,000 r/minute). HPLC-MS/MS was used to measure the metabolites of the probe substrates.

#### 2.5.4. Conditions of Ultra-Performance Liquid Chromatography (UPLC)-MS/MS

The UPLC-MS/MS system consisted of an Acquity UPLC device (Waters Corporation, Milford, MA, USA) and a triple quadruple mass spectrometer (Triple Quad 5500; Applied Biosystems, Foster City, CA, USA) equipped with an electrospray ionization source. The Acquity Waters BEH C18 (2.1 × 50 mm, 1.7 *μ*m) column was used. The mobile phases were as follows: water containing 0.1% formic acid and acetonitrile (mobile phase A) and 0.1% formic acid (mobile phase B). The gradient elution was as follows: 0 to 3 minutes (10 ⟶ 65%A), 3 to 3.5 minutes (65 ⟶ 90%A), and 3.5 to 4.5 minutes (90 ⟶ 10A%). The flow rate was 0.35 mL/minute, and the injection volume was 1 *μ*L.

For MS/MS detection, an electrospray ionization in a multireaction monitoring mode was operated with polarity switching between negative and positive ion modes. The mass spectrometer parameters were set as follows: source temperature, 120°C; capillary voltage, 3 kV; drying gas flow rate (N_2_), 1000 L/h; gas temperature, 600°C; collision gas, Ar; flow rate (Ar), 0.16 mL/min. The MRM analysis was conducted by monitoring the precursor ion to produce ion transitions of *m/z* 152 ⟶ 110 for acetaminophen, 362.2 ⟶ 214 for 5-hydroxyomeprazole, 305.3 ⟶ 269.3 for 6*β*-hydroxytestosterone, 183.8 ⟶ 120 for 6-hydroxychloroxazone, 285 ⟶ 186 for 5-hydroxytolbutamide, and 417.1 ⟶ 267.1 for puerarin.

#### 2.5.5. Changes in CYP450 Enzyme Activity in Different Groups of Mice

The corresponding mouse CYP450 enzymes, CYP450 isoenzyme probe substrates, and metabolites of probe substrates are shown in Table 2 [25–29]. The liver microsomes of the control, model, control HQD-3d, and model HQD-3d group were incubated with mixed probe substrates. Three parallel samples were set up in each group, and the production of the metabolites of probe substrates in each group was determined.

### 2.6. Effects of DN and HQD on the Expression of P450 Metabolic Enzymes and Small Intestine Transporters

Western blot was used to determine the relative protein expression of liver metabolic enzymes (Cyp1A2, Cyp2C37, Cyp3A11, Cyp2E1, and Cyp2C11) and small intestinal transporters (BCRP, P-gp, OCT1, OCT2, MRP1, and MRP2) in the control, model, control HQD-3d, and model HQD-3d groups. Membrane proteins of the liver and small intestine were harvested using a membrane protein extraction kit (Thermo Fisher Scientific), and the protein concentrations were determined using a BCA protein assay kit (Solarbio). Equal amounts of protein were added to loading buffer and resolved on 8% sodium dodecyl sulfate-polyacrylamide gel via electrophoresis. After transfer and blocking steps, membranes were incubated at 4°C for 12 hours with primary antibodies. Then, the membranes were incubated with corresponding secondary antibody for 2 hours. Subsequently, the membranes were incubated with ECL western blotting substrate for 1 minute and placed into the GelDoc XR gel documentation system (Bio-Rad Laboratories, Hercules, CA, USA) for photographing. Grayscale analysis was performed using Quantity-one (Bio-Rad Laboratories) to quantify the relative protein expression levels. GAPDH (Santa Cruz Biotechnology) was used to verify equal protein loading.

## 3. Results

### 3.1. Effects of DN and HQD on the Activity of Liver Metabolic Enzymes

Compared to the control group, the activity of Cyp2C11 and Cyp3A11 in the model group and Cyp2C11 in the control HQD-3d group was increased (Figure 2). The activities of Cyp1A2, Cyp2E1, Cyp3A11, and Cyp2C37 in the control HQD-3d group were decreased. Compared to the model group, the activities of Cyp1A2, Cyp3A11, and Cyp2C37 in the model HQD-3d group were decreased, while those of Cyp2C11 and Cyp2E1 were increased. DN induced the activity of Cyp2C11 and Cyp3A11. HQD inhibited the activity of Cyp1A2, Cyp2C37, Cyp3A11, and induced the activity of Cyp2C11. However, HQD inhibited the activity of Cyp2E1 in the control group, and induced the activity of Cyp2E1 in the model group. The results are shown in Figure 2 and Table 3.

### 3.2. Effects of DN and HQD on the Expression of Liver Metabolic Enzymes and Small Intestine Transporters

#### 3.2.1. Effect of DN on the Expression of Liver Cyp450 Enzymes and Small Intestinal Transporters

The effects of DN on the expression of liver Cyp450 enzymes and small intestinal transporters are summarized in Table 3. Compared to normal mice, expression of Cyp1A2 and Cyp2E1 in DN mice was decreased, and the expression of Cyp2C11 and Cyp2C37 was increased, but there was no significant difference (Figure 3). The activity of each Cyp450 enzyme was consistent with the expression results. Compared to normal mice, the expression of P-gp and BCRP in DN mice was significantly lower, whereas the expression of OCT1, OCT2, MRP1, and MRP2 was significantly increased (*P* < 0.001) (Figure 4). The results showed that the functions of Cyp450 enzymes and transporters changed in the state of DN. DN induced the expression of Cyp2C11, Cyp2C37, OCT1, OCT2, MRP1, and MRP2, and inhibited the expression of Cyp1A2, Cyp2E1, P-gp, and BCRP.

#### 3.2.2. Effects of HQD on the Expression of Liver Cyp450 Enzymes and Small Intestinal Transporters

The effects of HQD on the expression of liver Cyp450 enzymes and small intestinal transporters are shown in Table 3. Relevant western blots are also shown in Figure 3. As the clinical therapy requires long-term oral administration, in this experiment, animals were given multiple oral doses of the therapy. After 3 days of continuous administration, the effects of HQD on the expression of Cyp450 enzymes and intestinal transporters in normal and model mice were investigated. Compared to the control group, the expression of Cyp1A2 and Cyp3A11 in the control HQD-3d group was decreased significantly, and the expression of Cyp2E1 and Cyp2C37 tended to decrease, but there was no significant difference. Compared to the model group, the expression of Cyp2C37 and Cyp3A11 in the model HQD-3d group was decreased significantly, and while the expression of Cyp2E1 tended to increase, there was no significant difference. The activity of each Cyp450 enzyme was consistent with the expression result. Oral administration of HQD resulted in decreased expression of Cyp2C37 and Cyp3A11 in DN mice and decreased expression of Cyp1A2 and Cyp3A11 in normal mice.

The relevant western blots of small intestinal transporters are shown in Figure 4. Compared to the control group, the expression of intestinal transporters BCRP and P-gp in the control HQD-3d group was increased significantly, but the expression of OCT1, OCT2, MRP1, and MRP2 were unchanged. Compared to the model group, the expression of BCRP in the model HQD-3d group was increased significantly, while the expression of OCT2, MRP1, and MRP2 was decreased, and OCT1 and P-gp were unchanged. These results suggest that HQD stimulates the expression of BCRP and P-gp in normal mice, and BCRP in DN mice. Conversely, HQD inhibits the expression of OCT2, MRP1, and MRP2 in DN mice. The regulatory effects of HQD on some liver metabolic enzymes and transporters under physiological and pathological conditions are different.

## 4. Discussion

Liver CYP450s enzymes are involved in the metabolism of approximately 90% of clinical drugs [30], including CYP1, CYP2, and CYP3. Among them, 1A2, 2C19, 3A4, 2E1, 2C9, and 2D6 are the six main subtypes of CYP450, accounting for approximately 80% of the total CYP450 enzymes in the liver [31]. In pilot studies, we found that the main active ingredients of HQD (astragaloside IV, calycosin-glucuronide, formononetin, and glycyrrhizic acid) may be metabolized by Cyp1A2, 2C19, 3A4, 2E1, and 2C9 (data unpublished). Therefore, 1A2, 2C19, 3A4, 2E1, and 2C9 were chosen for this study. Although CYP450 subtypes are species and genera-specific, they also have lineal homology and similar functions. Mouse Cyp1A2, 2C37, 3A11, 2E1, and 2C11 are homologous to human CYP1A2, 2C19, 3A4, 2E1, and 2C9, respectively [28, 29].

In the small intestine, transporters modulate the efflux and influx of exogenous and endogenous substances. Through controlling the cell transit of orally ingested substances, the transport enzyme system mediates drug bioavailability [32]. Of clinical relevance, the function and expression of drug transporters are altered in disease, which affect the treatment effects and pharmacokinetics. Clarifying the transport mechanism could improve the safety and effectiveness of drugs and improve clinical usage. Intestinal efflux transporters (e.g., P-gp, BCRP, and MRP) can have varied activities depending on the local balance between drug effect and overlap with other agents [33, 34]. Previous studies showed that the efflux of flavonoids and glucuronic acid metabolites contributes to their low bioavailability. In the intestine, flavonoids and glucuronide metabolites are excreted into the intestinal lumen by efflux transporters (i.e., P-gp, BCRP, and MRP2). For example, calycosin-7-O-*β*-D-glucoside is hydrolyzed into aglycon by hydrolase in the intestine. The generated metabolites can then be transported into the intestinal lumen by efflux transporters (BCRP or MRP2) [35].

When any drug is administered alone, the presence of chronic disease such as diabetes and subsequent DN is predicted to dominate drug availability. Changes in the expression levels of P-gp, BCRP, and MRP2 cause changes in the pharmacokinetic process of calycosin-7-O-*β*-D-glucoside, ononin, and the metabolites of aglycones. Glycyrrhizic acid can affect the function of P-gp on Caco-2 in the cell membrane, regulate P-gp-mediated drug efflux, and alter P-gp-mediated efflux, thus changing drug pharmacokinetics [36, 37]. Data indicated that P-gp inhibitors increased the efficacy and bioavailability of astragaloside IV, suggesting that astragaloside IV is a substrate of P-gp [38]. Changes in the expression levels of P-gp may account for altered *in vivo* pharmacokinetics of astragaloside IV and glycyrrhizic acid. Moreover, owing to the limited studies on OCT_s,_ whether the up-regulation of OCT1 and OCT2 expression in DN is a factor in pharmacokinetic changes needs to be confirmed by further research.

In a single dose, we mainly consider the influence of pathological factors on drugs. Compared to normal mice, the expression of P-gp and BCRP in DN mice was significantly lower (*P* < 0.05 and *P* < 0.001); the activity and expression of Cyp2C11, Cyp3A11, and Cyp2C37 in DN mice was increased, while that of Cyp1A2 and Cyp2E1 was decreased. Drugs absorbed and excreted through the small intestine can also be metabolized by Cyp450s in the liver. The dual mediating effect of Cyp450s and the intestinal efflux transporter determines the speed and degree of drug absorption. Compared to the effect of Cyp2C11, Cyp3A11, and Cyp2C37, we speculate that the changes in pharmacokinetic parameters of HQD in DN may be mainly mediated by the down-regulation of P-gp and BCRP expression, which results in an increase in the AUC and a decrease in the CL_Z/F_ of astragaloside IV, glycyrrhizic acid, calycosin-7-O-*β*-D-glucoside, ononin, and the metabolites of aglycones.

TCMs may inhibit or induce the expression of small intestine transporters, thus affecting the *in vivo* disposal of substrates. The results of the present study found that HQD increased expression of BCRP in normal and DN mice, increased expression of P-gp in normal mice, and inhibited expression of OCT2, MRP1, and MRP2 in DN mice. Therefore, the actions of HQD upon transporter expression levels were dependent upon the health status of the animals.

HQD inhibits the activity of Cyp1A2, Cyp2C37, and Cyp3A11, and induces the activity of Cyp2C11 in diabetic mice. Of relevance, many diabetes drugs are metabolized by CYP2C9, CYP3A4, and CYP2C8 [39]. For example, sulfonylurea hypoglycemics are metabolized by CYP2C9 and CYP3A4. Inhibition or induction of these enzymes will alter drug metabolism and likely increase plasma concentrations, which in turn may disturb the glucose balance [40, 41]. Together, our data underscore the need to employ HQD with caution in diabetic individuals, especially in the presence of chronic renal disease.

CYP450 enzymes participate in the synthesis and metabolism of bile and fatty acids and steroids. Changes in liver CYP450 enzymes and intestinal transporters have been noted in diabetes [42, 43]. In diabetics, testosterone, estradiol, and retinoic acid levels are decreased [44–47], suggesting a possible need for supplementation of testosterone, estradiol, and retinoic acid. Of note, testosterone, estradiol, and retinoic acid are metabolized by CYP3A4 [48]. We found that Cyp3A11 activity was increased in the model group but was decreased after HQD treatment. Mouse Cyp3A11 is homologous to human CYP3A4, and its function is similar [31]. It is thus expected that HQD will, via inhibition of CYP3A4, reduce elimination of testosterone, estradiol, and retinoic acid.

## 5. Conclusion

HQD altered protein levels and activity of multiple liver enzymes and intestinal epithelial transport molecules in a disease-dependent manner. Further, in animal DN, changes in HQD pharmacokinetics were linked to decreased expression of P-gp and BCRP. These data provide additional insights into the safe usage of HQD in health and DN. However, whether the six active ingredients (astragaloside IV, calycosin-7-O-*β*-D-glucoside, calycosin-glucuronide, ononin, formononetin, and glycyrrhizic acid) of HQD are transport substrates for P-gp and BCRP needs to be confirmed by further research.

## Figures and Tables

**Figure 1:** The HPLC-MS/MS chromatogram of HQD. Blank sample (a), reference substance of six active ingredients in HQD (b), and HQD sample (c). (1) astragaloside IV, (2) calycosin-7-O-*β*-D-glucoside, (3) calycosin-glucuronide, (4) ononin, (5) formononetin, (6) glycyrrhizic acid, (7) puerarin (IS), (8) digoxin (IS).

**Figure 2:** The number of metabolites produced by specific probe substrates in liver microsomes (*μ*mol/mL, *x* ± SD, *n* = 6). ^*∗*^*P* < 0.05, ^*∗∗*^*P* < 0.01, ^*∗∗∗*^*P* < 0.001 compared to the control group; ^#^*P* < 0.05, ^##^*P* < 0.01, ^###^*P* < 0.001 compared to the model group.

**Figure 3:** Protein expression of CYP450 metabolic enzymes (Cyp1A2, Cyp2C37, Cyp3A11, Cyp2E1, and Cyp2C11) in different groups (*n* = 3). ^*∗*^*P* < 0.05, ^*∗∗*^*P* < 0.01, ^*∗∗∗*^*P* < 0.001 compared to the control group; ^#^*P* < 0.05, ^##^*P* < 0.01, ^###^*P* < 0.001 compared to the model group.

**Figure 4:** Protein expression of small intestinal transporters (BCRP, P-gp, OCT1, OCT2, MRP1, and MRP2) in different groups (*n* = 3). ^*∗*^*P* < 0.05, ^*∗∗*^*P* < 0.01, ^*∗∗∗*^*P* < 0.001 compared to the control group; ^#^*P* < 0.05, ^##^*P* < 0.01, ^###^*P* < 0.001 compared to the model group.

**Table 1:** Content of each component extracted from three batches of *Astragalus* and *Glycyrrhizae* (*x* ± SD, *n* = 3).

Extraction fraction	Constituents	Content (%)	Assay methods
Astragalus saponins extract	Astragalus saponins	72.97 ± 1.06	Ultraviolet-visible spectrophotometer (UV)
	Astragaloside IV	2.72 ± 0.10	High performance liquid chromatography (HPLC)
Astragalus flavones extract	Astragalus flavones	70.58 ± 2.16	UV
	Calycosin-7-O-*β*-D-glucoside	1.67 ± 0.08	HPLC
	Calycosin-glucuronide	1.45 ± 0.10	HPLC
	Ononin	0.91 ± 0.09	HPLC
	Formononetin	0.32 ± 0.02	HPLC
Astragalus polysaccharides extract	Astragalus polysaccharides	67.12 ± 2.60	UV
Glycyrrhizic acid extract	Glycyrrhizic acid	81.02 ± 1.04	HPLC

**Table 2:** Substrates and metabolites of CYP450 enzymes.

Human liver CYP450 enzyme	Corresponding mouse CYP450 enzymes	Probe substrates	Metabolites
CYP1A2	Cyp1A2	Phenacetin	Acetaminophen
CYP2C19	Cyp2C37	Omeprazole	5-hydroxyomeprazole
CYP3A4	Cyp3A11	Testosterone	6*β*-hydroxytestosterone
CYP2E1	Cyp2E1	Chlorzoxazone	6-hydroxychloroxazone
CYP2C9	CypC11	Tolbutamide	5-hydroxytolbutamide

**Table 3:** Changes in CYP450s and transporter enzymes after oral administration of HQD.

No.	CYP450s and transporter	Model vs. Control		Control HQD-3d		Model HQD-3d vs. Model	
		Activity	Expression	*V* Control		Activity	Expression
				Activity	Expression		
1	Cyp1A2	↓	↓	↓^*∗∗*^	↓^*∗*^	↓^##^	—
2	Cyp2C11	↑^*∗∗∗*^	↑	↑^*∗∗*^	—	↑^##^	—
3	Cyp2C37	↑	↑	↓^*∗∗*^	↓	↓^###^	↓^#^
4	Cyp2E1	↓	↓	↓^*∗∗∗*^	↓	↑^##^	↑
5	Cyp3A11	↑^*∗∗*^	—	↓^*∗*^	↓^*∗∗*^	↓^###^	↓^##^
6	BCRP	—	↓^*∗∗∗*^	—	↑^*∗∗*^	—	↑^##^
7	P-gp	—	↓^*∗*^	—	↑^*∗∗∗*^	—	—
8	OCT1	—	↑^*∗∗∗*^	—	—	—	—
9	OCT2	—	↑^*∗∗∗*^	—	—	—	↓^#^
10	MRP1	—	↑^*∗∗∗*^	—	—	—	↓^###^
11	MRP2	—	↑^*∗∗∗*^	—	—	—	↓^#^

^*∗*^ *P* < 0.05, ^*∗∗*^*P* < 0.01, ^*∗∗∗*^*P* < 0.001 compared to the control; ^#^*P* < 0.05, ^##^*P* < 0.01, ^###^*P* < 0.001 compared to the model; no obvious trend “—”.

## Data Availability

The data used to support the findings of this study are available from the corresponding author upon reasonable request.
